The article "The Variation of Nasal Microbiota Caused by Low Levels of Gaseous Ammonia Exposure in Growing Pigs" was retracted in 2025. Reasons: unreliable results or conclusions; concerns about the article.

# The Variation of Nasal Microbiota Caused by Low Levels of Gaseous Ammonia Exposure in Growing Pigs

**DOI:** 10.3389/fmicb.2019.01083

**Published:** 2019-05-16

**Authors:** Tongxin Wang, Qiongyu He, Weilei Yao, Yafei Shao, Ji Li, Feiruo Huang

**Affiliations:** Department of Animal Nutrition and Feed Science, College of Animal Science and Technology, Huazhong Agricultural University, Wuhan, China

**Keywords:** nasal microbiota, gaseous ammonia exposure, growing pigs, growth performance, respiratory tract

## Abstract

Exposure to gaseous ammonia, even at low levels, can be harmful to pigs and human health. However, less is known about the effects of sustained exposure to gaseous ammonia on nasal microbiota colonization in growing pigs. A total of 120 Duroc×Landrace×Yorkshire pigs were housed in 24 separate chambers and continuously exposed to gaseous ammonia at 0,5, 10, 15, 20, and 25 ppm (four groups per exposure level) for 4 weeks. Then, we used high-throughput sequencing to perform 16S rRNA gene analysis in nasal swabs samples from 72 pigs (*n* = 12). The results of the nasal microbiota analysis showed that an increase in ammonia concentration, especially at 20 and 25 ppm, decreased the alpha diversity and relative abundance of nasal microbiota. *Proteobacteria, Firmicutes, Bacteroidetes, Actinobacteria*, and *Chloroflexi* were the most abundant phyla. In addition, the relative abundances of 24 microbial genera significantly changed as the ammonia level increased. Four microbial genera (*Pseudomonas, Lactobacillus, Prevotella*, and *Bacteroides*) were significantly decreased at 25 ppm, while only two genera (*Moraxella* and *Streptococcus*) were increased at 25 ppm. PICRUSt analyses showed that the relative abundances of the nasal microbiota involved in cell motility, signal transduction, the nervous system, environmental adaptation, and energy and carbohydrate metabolism were significantly decreased, while genes involved in the immune system, endocrine system, circulatory system, immune system diseases and metabolism of vitamins, lipid, and amino acids were increased with increased ammonia levels. The results of *in vivo* tests showed that an increase in ammonia levels, especially an ammonia level of 25 ppm, caused respiratory tract injury and increase the number of *Moraxella* and *Streptococcus* species, while simultaneously decreasing respiratory immunity and growth performance, consistent with the increased presence of harmful bacteria identified by nasal microbiota analysis. Herein, this study also indicted that the threshold concentration of ammonia in pig farming is 20 ppm.

## Introduction

The intensive feeding of pigs continuously exposes pigs to high concentrations of aerial pollutants, such as organic dust, noxious gases, microorganisms, and bacterial endotoxins, which greatly causes subclinical disease and production losses (Aarnink et al., 1995; Liu et al., 2017). As one of the most important gaseous pollutants in pig sheds, ammonia is produced through the decomposition of animal droppings in the presence of microorganisms under heat and moisture conditions (Xiong et al., 2016). For decades, ammonia emission has received increasing attention for its potential negative impacts on farming environments, the ecosystem, and human and animal health (Murphy et al., 2012; Costa, 2017).

The article "The Variation of Nasal Microbiota Caused by Low Levels of Gaseous Ammonia Exposure in Growing Pigs" was retracted in 2025. Reasons: unreliable results or conclusions; concerns about the article.

It is generally accepted that gaseous ammonia at high levels is a severe respiratory tract irritant capable of inhibiting the efficiency of the respiratory system (Smith et al., 1996). However, even low concentrations of ammonia, such as 10 or 15 ppm, still have adverse effects on the health of pigs, potentially causing atrophic rhinitis and respiratory disease (Hamilton et al., 1998; Michiels et al., 2015). Recently, it was reported that the microbial populations of the upper respiratory tract of pigs had a close association with respiratory diseases (Lanaspa et al., 2017). Besides, the nose is one of the main interfaces between the internal body and the external environment, and it is the first microbial barrier to infection. In addition, the nose can harbor important microorganisms that can be pathogenic under certain circumstances (Correa-Fiz et al., 2016). A previous study about fecal and nasal microbiotas of pigs during early life demonstrated that the gastrointestinal and respiratory tracts are exposed to thousands of bacteria species with significant turnover in community membership and structure until a relative degree of stability is evident at 2–3 weeks post-weaning (Slifierz et al., 2015). Another study indicated that nasal bacterial communities have a close relationship with the occurrence of Glässer's disease in pigs (Correa-Fiz et al., 2016). Therefore, studies on nasal microbiota can be relevant.

There has been a great interest in a recent study on nasal microbiota using pigs as models due to their similarities to human beings in relation to airborne microbial communities (Kraemer et al., 2018). In addition, the respiratory tracts of farmers also receive much attention and has been shown to be very affected by pig farming (Oppliger et al., 2012; Wardyn et al., 2015). It was found that the nasal microbiota of pig farmers was similar to that of pigs, suggesting animal-human microbial transmission within pig farms and that the air environment influences animals and humans in a similar manner (Kraemer et al., 2018). Considering that ammonia concentrations on pig farms are not extremely high, the legal exposure level for humans in Ohio piggeries was 25 ppm (Costa et al., 2003). However, even low levels of gaseous ammonia have toxic effects on the respiratory tract of pigs and humans. Thus, elucidating the effect of low levels of gaseous ammonia on the nasal microbiota composition in pigs is of great interest.

The article "The Variation of Nasal Microbiota Caused by Low Levels of Gaseous Ammonia Exposure in Growing Pigs" was retracted in 2025. Reasons: unreliable results or conclusions; concerns about the article.

Here, the aims of this article are to reveal the nasal microbiota compositions and functional maturation of nasal bacterial communities in piglets exposed to different low levels of gaseous ammonia, by using the environmentally controlled chambers (Timbrell et al., 1970), we analyzed the nasal microbiota of 72 pigs exposed to different low levels of gaseous ammonia, and also the respiratory mucosal barrier, and growth performance, then we suggest the threshold concentration of ammonia for pig farming and discuss the potential relationship between nasal microbiota variations and respiratory health of growing pigs under low concentrations of ammonia.

## Materials and Methods

### Ammonia Treatment and Environmental Chamber Parameters

The animal handling protocol (permit number: HZAUSW2017-0006) followed in this study was approved by the Animal Care and Use Committee of College of Animal Sciences and Technology, Huazhong Agricultural University and was in compliance with the National Research Council's Guide for the Care and Use of Laboratory Animals. The methods were carried out in accordance with the approved guidelines. The Hubei Jinlin animal company approved the animal studies. One hundred and twenty castrated Duroc × Landrace × Yorkshire pigs weighing ~30.2 ± 1 kg were equally housed for a total of 4 weeks in twenty 2.5 m^3^ environmentally controlled chambers with free access to feed and drinking water (Timbrell et al., 1970). The chambers were set for 6 different gaseous ammonia concentrations (0, 5, 10, 15, 20, and 15 ppm), 20 pigs per exposure level (4 separate chambers per exposure level, 5 pigs per chambers). All chambers were in the same pigsty. The amount of ammonia gas was determined after preliminary debugging. The mixture of ammonia gas and the pumping of fresh air into the is pigsty was determined by an ammonia gas sensor with an accuracy of 0.1 ppm. To control the influence of feces and urine on the production of harmful gases, feces, and urine was removed hourly through a defecation device in the drainage channel. The ammonia concentration in the box was guaranteed to reach the set value, and the influence of other harmful gases on the test was basically eliminated. Combined with an optical ammonia sensor, the environmental ammonia parameters in the box were recorded in 24 h increments (major equipment is shown in Figure S1). Within each chamber, the air was maintained at a temperature of 25 ± 1.0°C, with a relative humidity of 65 ± 5% and an air flow speed of 0.2 m/s.

The article "The Variation of Nasal Microbiota Caused by Low Levels of Gaseous Ammonia Exposure in Growing Pigs" was retracted in 2025. Reasons: unreliable results or conclusions; concerns about the article.

All experimental pigs were given water *ad libitum* and fed twice a day using corn-soybean-based diets (Dabeinong Company, Wuhan, China) containing 0.61% calcium, 0.6% phosphorus, 17% crude protein, 1,380 kJ digestible energy and 0.85% lysine. The average daily gain (ADG), average daily feed intake (ADFI), and feed conversation ratio (FCR) were determined by weighing pigs and measuring feed consumption every 7 d. The piglets with clinical symptoms, such as coughing, sneezing, difficult breathing and conjunctivitis, were observed every 7 d. Nasal swabs were taken from the nares of 72 animals (*n* = 12) after 28 d of exposure and placed into sterile tubes. Swabs were transported to the laboratory on ice where they were resuspended in 500 μl of PBS and stored at −20°C for further microbial analysis. The animals (72 pigs, 12 pigs per exposure level) were sacrificed after 28 d of exposure. Blood was collected from the precaval vein, and lung and trachea samples were collected for histological analysis (after animals were sacrificed). All animals were healthy and did not receive any antibiotic treatment before slaughter, and the pigs were sacrificed by administering a pentobarbital overdose after monitoring was finished.

### Microbial Genomic DNA Extraction

Total bacterial genomic DNA was extracted using FastDNA SPIN extraction kits (MP Biomedicals, Santa Ana, CA, USA) following the manufacturer's instructions and stored at −20°C until further analysis. The quantity and quality of extracted DNA were measured using a NanoDrop ND-1000 spectrophotometer (Thermo Fisher Scientific, Waltham, MA, USA) and agarose gel electrophoresis, respectively.

### 16S rDNA Amplicon Pyrosequencing

PCR amplification of the bacterial 16S rRNA genes V3–V4 region was performed using the forward primer 338F (5′-ACTCCTACGGGAGGCAGCA-3′) and the reverse primer 806R (5′-GGACTACHVGGGTWTCTAAT-3′). Sample -specific 7-bp barcodes were incorporated into the primers for multiplex sequencing. The PCR components contained 5 μl of Q5 reaction buffer (5 ×), 5 μl of Q5 High-Fidelity GC buffer (5 ×), 0.25 μl of Q5 High-Fidelity DNA Polymerase (5U/μl), 2 μl (2.5 mM) of dNTPs, 1 μl (10 μM) of each Forward and Reverse primer, 2 μl of DNA Template, and 8.75 μl of ddH_2_O. Thermal cycling consisted of initial denaturation at 98°C for 2 min, followed by 25 cycles consisting of denaturation at 98°C for 15 s, annealing at 55°C for 30 s, and extension at 72°C for 30 s, with a final extension of 5 min at 72°C. PCR amplicons were purified with Agencourt AMPure Beads (Beckman Coulter, Indianapolis, IN) and quantified using the PicoGreen dsDNA Assay Kit (Invitrogen, Carlsbad, CA, USA). After the individual quantification step, amplicons were pooled in equal amounts, and pair-end 2 × 300 bp sequencing was performed using the Illlumina MiSeq platform with MiSeq Reagent Kit v3 at Shanghai Personal Biotechnology Co., Ltd (Shanghai, China).

The article "The Variation of Nasal Microbiota Caused by Low Levels of Gaseous Ammonia Exposure in Growing Pigs" was retracted in 2025. Reasons: unreliable results or conclusions; concerns about the article.

### Sequence Analysis

The Quantitative Insights Into Microbial Ecology (QIIME, v1.8.0) pipeline was employed to process the sequencing data, as previously described (Caporaso et al., 2010). Briefly, raw sequencing reads with exact matches to the barcodes were assigned to respective samples and identified as valid sequences. The low-quality sequences were filtered through following criteria (Gill and Nelson, 2006; Chen and Jiang, 2014): sequences that had a length of <150 bp, sequences that had average Phred scores of <20, sequences that contained ambiguous bases, and sequences that contained mononucleotide repeats of >8 bp. Paired-end reads were assembled using FLASH (v1.2.7) (Magoc and Salzberg, 2011). After chimera detection, the QIIME software (v1.8.0) call USEARCH (v5.2.236) check and remove chimeric sequences the remaining high-quality sequences were clustered into operational taxonomic units (OTUs) at 97% sequence identity by UCLUST (v1.2.22q) (Edgar, 2010). A representative sequence was selected from each OTU using default parameters. OTU taxonomic classification was conducted by BLAST searching the representative sequences set against the Greengenes Database (Desantis et al., 2006) using the best hit (Altschul et al., 1997). An OTU table was further generated to record the abundance of each OTU in each sample and the taxonomy of these OTUs. OTUs containing <0.001% of total sequences across all samples were discarded. To minimize the difference of sequencing depth across samples, an averaged, rounded rarefied OTU table was generated by averaging 100 evenly resampled OTU subsets under the 90% of the minimum sequencing depth for further analysis.

### Biochemical Assays and Histological Analysis

The levels of blood ammonia, blood urea nitrogen (BUN), superoxide dismutase (SOD), total antioxidant capacity (T-AOC), lactate dehydrogenase (LDH), and aspartate aminotransferase (AST) in serum, and IgA, IgG, and IgM in the trachea were determined using commercial assay kits (Sigma) according to the manufacturer's protocol. For the histological examination, tracheal, and lung tissues were collected and fixed in 10% neutral buffered formalin and embedded in paraffin. Standard 5 μm thickness sections were cut, stained with hematoxylin and eosin (H&E) and examined by light microscopy (Chaudhari et al., 2012).

The article "The Variation of Nasal Microbiota Caused by Low Levels of Gaseous Ammonia Exposure in Growing Pigs" was retracted in 2025. Reasons: unreliable results or conclusions; concerns about the article.

Reverse Transcriptase-Polymerase Chain Reaction (RT-PCR) analysis

Total RNA was extracted from trachea using TRIzol reagent; it was converted to cDNA by reverse transcription. The sequences of trachea-related gene primers (sense and anti-sense) were used for the generation of cDNAs:

gapdh-S, 5′-GTGAAGGTCGGAGTGAACGGA-3′

gapdh-A, 5′-CCATTTGATGTTGGCGGGAT-3′

CLAUDIN-1-S, 5′-CCCGTGCCTTGATGGTAATTG-3′

CLAUDIN-1-A 5′-AAAGTAGGGCACCTCCCAGAAG-3′

CASP3-S 5′-GGAAGCAAATCAATGGACTCTG-3′

CASP3-A 5′-TGCTCCTTTTGCTATGGTCTTCT-3′

MUC5B-S 5′-ACAACGCCCTCAACGACTTCA-3′

MUC5B-A 5′-GGTGGAGTCAACCTGAGAACG-3′

PCR products were run on 2% agarose gels, stained with ethidium bromide and photographed.

### Real-Time PCR Assay for Microbiota Quantification From Nasal Swabs of Piglets

Real-time PCR was performed on an iCycler IQ real-time detection system associated with the iCycler optical system interface software version 2.3 (Bio-Rad, Veenen-daal, the Netherlands). The amount of DNA in each treatment was determined, and the mean values were calculated. A standard curve was generated using serially diluted 16 S rRNA gene amplicons obtained from the species-specific primer *Moraxella catarrhalis* UspA1 (Tao et al., 2017) and used for the quantification of *Moraxella catarrhalis*. PCR was performed under following conditions: initial DNA denaturation at 95°C for 10 min, followed by 35 cycles of denaturation at 95°C for 45 s, and primer annealing and extension at 72°C for 10 min. Total *Streptococcus pneumoniae* were quantified using the following PCR program: 3 min at 95°C, 20 s at 95°C, followed by 40 cycles of 15 s at 72°C and 10 min at 72°C (56).

### Bioinformatics and Statistical Analysis

Sequence data analyses were mainly performed using QIIME and R packages (v3.2.0). OTU-level alpha diversity indices, such as Chao1 richness estimator, ACE metric (Abundance-based Coverage Estimator), Shannon diversity index, and Simpson index, were calculated using the OTU table in QIIME. OTU-level ranked abundance curves were generated to compare the richness and evenness of OTUs among samples. Beta diversity analysis was performed to investigate the structural variation of microbial communities across samples using UniFrac distance metrics (Lozupone and Knight, 2005; Lozupone et al., 2007) and visualized via principal coordinate analysis (PCoA), non-metric multidimensional scaling (NMDS) and unweighted pair-group method with arithmetic means (UPGMA) hierarchical clustering (Ramette, 2010). Differences in the Unifrac distances for pairwise comparisons among groups were determined using Student's *t*-test and the Monte Carlo permutation test with 1,000 permutations, and visualized through the box-and-whiskers plots. Principal component analysis (PCA) was also conducted based on the genus-level compositional profiles (Ramette, 2010). The significance of differentiation of microbiota structure among groups was assessed by PERMANOVA (Permutational multivariate analysis of variance) (Mcardle and Anderson, 2001) and ANOSIM (Analysis of similarities) (Clark et al., 1993; Warton et al., 2012) using R package “vegan.” The taxonomy compositions and abundances were visualized using MEGAN (Huson et al., 2011) and GraPhlAn (Asnicar et al., 2015). Venn diagram was generated to visualize the shared and unique OTUs among samples or groups using R package “Venn Diagram,” based on the occurrence of OTUs across samples/groups regardless of their relative abundance (Zaura et al., 2009). Taxa abundances at the phylum, class, order, family, genus levels were statistically compared among samples or groups by Metastats (White et al., 2009; Parks et al., 2014), and visualized as violin plots. LEfSe (Linear discriminant analysis effect size) was performed to detect differentially abundant taxa across groups using the default parameters (Segata et al., 2011). PLS-DA (Partial least squares discriminant analysis) was also introduced as a supervised model to reveal the microbiota variation among groups, using the “plsda” function in R package “mixOmics” (Chen et al., 2011). Random forest analysis was applied to discriminating the samples from different groups using the R package “randomForest” with 1,000 trees and all default settings (Breiman, 2001; Liaw and Wiener, 2002). The generalization error was estimated using 10-fold cross-validation. The expected “baseline” error was also included, which was obtained by a classifier that simply predicts the most common category label. Co-occurrence analysis was performed by calculating Spearman's rank correlations between predominant taxa. Correlations with |RHO| > 0.6 and *P* < 0.01 were visualized as co-occurrence network using Cytoscape (Shannon et al., 2003). Microbial functions were predicted by PICRUSt (Phylogenetic investigation of communities by reconstruction of unobserved states), based on high-quality sequences (Langille et al., 2013). Results of respiratory mucosal barrier, growth performance analyses were conducted using Prism5 (Graph Pad Software). The results are expressed as the means ± SD. Data were compared with a two -way ANOVA with a subsequent Bonferroni *post-test* for multiple comparisons or with Student's *t*-test. For all tests, *P* < 0.05 was considered significant.

The article "The Variation of Nasal Microbiota Caused by Low Levels of Gaseous Ammonia Exposure in Growing Pigs" was retracted in 2025. Reasons: unreliable results or conclusions; concerns about the article.

## Results

### 16s RDNA Sequence Data From the Nasal Microbiota of Growing Pigs Under Low Levels of Gaseous Ammonia Exposure

To investigate the nasal microbiota of pigs under different low levels of gaseous ammonia exposure, this study used chambers with a wireless gas sensor system that was able to accurately automatically control the gaseous ammonia concentrations. The height of the ammonia sensor installation was consistent with the standing height of growing pigs; after the concentration of ammonia reached the set concentration in the mixing air box, it was passed into the box to control the ammonia concentration accurately. We amplicon-sequenced nasal swab samples from the growing pigs at 6 ammonia levels (0, 5, 10, 15, 20, and 25 ppm) in each chamber and collected a total of 2,815,214 high-quality sequences from 72 pig swabs (*n* = 12). Rarefaction curves demonstrated that almost all microbial species were detected in the nasal fluid of growing pigs (Figure 1A).

**Figure 1:** Nasal microbial OTUs development under low levels of gaseous ammonia exposure. **(A)** Microbial rarefaction curves based on Chao index (description and sample ID) were used to assess the depth of coverage for each sample. Each treatment samples were distinguished by different colors of lines. **(B,C)** Venn diagrams for Microbial OTUs compositions.

Based on 97% sequence similarity, all the sequences were clustered into 15868 OTUs, and the Venn diagrams are shown in Figures 1B,C. The OTUs were classified into 6 phyla. No significant differences were observed among the OTUs from samples exposed to 0, 5, 10, and 15 ppm, while the numbers of OTUs from samples exposed to 20 and 25 ppm were significantly lower than those in the other groups.

### Alterations in Nasal Microbial Diversities With the Low Levels of Gaseous Ammonia Exposure

To analyze the dynamics of nasal microbial communities during low levels of gaseous ammonia exposure, we evaluated the alpha diversity of the microbial communities. The results of the Chao index, Shannon index, ACE index and Simpson index are shown in Figure 2. The indices that reflect species richness and evenness were all shown to be significantly decreased with the increase in ammonia concentrations ranging from 0 to 25 ppm. Interestingly, no significant differences were observed in the indices ranging from 0 to 15 ppm, while all the indices of samples exposed to 20 and 25 ppm were significantly lower than those in the other groups (*p* < 0.05) (Figures 2A–D). These results indicated that the alpha diversity of the nasal microbial community was significantly decreased in samples exposed to concentrations of 20–25 ppm ammonia.

The article "The Variation of Nasal Microbiota Caused by Low Levels of Gaseous Ammonia Exposure in Growing Pigs" was retracted in 2025. Reasons: unreliable results or conclusions; concerns about the article.

**Figure 2:** The changes of nasal microbial diversities with the low levels of gaseous ammonia exposure. **(A)** Microbial alpha diversity determined by Chao index. **(B)** Microbial alpha diversity determined by Shannon index. **(C)** Microbial alpha diversity determined by ACE index. **(D)** Microbial alpha diversity determined by Simpson index. **(E)** Scatterplot from PCoA, based on unweighted UniFrac distance in microbial communities. **(F)** Scatterplot from PCoA, based on weighted UniFrac distance in microbial communities. Different letters above the bars denotes a significantly different alpha diversity index among groups.

To further understand the differences among the microbiota from nasal samples, the beta diversity was estimated. Weighted and unweighted UniFrac phylogenetic distances were used to generate beta diversity distance matrices and calculate the degree of differentiation among the samples. Principal coordinate analysis (PCoA) was performed for each group, and resampling was performed repeatedly on a subset of the available data of each sample evenly to measure the robustness of individual clusters in the PCoA plots. The emperor PCoA plots obtained are depicted in Figures 2E,F. The R^2^ was measured to test for the percentage of variation among samples in each group using Adonis, a non-parametric statistical method, in the Vegan package of R (Caporaso et al., 2010). The mean distances among the six groups (0–25 ppm) were calculated and were shown to be significantly different in the unweighted analysis (*R*^2^ = 0.6904, *p* = 0.001), indicating a qualitatively different composition of the microbiota according to the increase in the ammonia concentration. The weighted analysis also showed differences in the composition of the microbiota from samples exposed to different ammonia concentrations (*R*^2^ = 0.5748, *p* = 0.002), showing a significantly different composition of microbiota among the groups. Both of the UniFrac phylogenetic distances showed that when the pigs were exposed to gaseous ammonia at 25 ppm, the distances were significantly different from the other groups (Figures 2E,F).

### Alterations in Nasal Microbial Taxonomic Compositions Associated With Low Levels of Gaseous Ammonia Exposure

After the microbial OTU representative sequences were taxonomically classified, differences at several taxonomic levels were found in the nasal microbiota composition of piglets exposed to different low levels of gaseous ammonia. The relative abundances of six different taxonomic levels is shown in Figure 3 (phylum and genus) and Figure S2 (class, order, and family) (each OTU presents the mean value for the 12 pigs, *n* = 12). The results showed that *Proteobacteria* constituted ~36.4% of the total sequences on average and was the most abundant phylum. The second most abundant phylum, *Firmicutes*, constituted ~34.8% of the total sequences on average, followed by the phyla *Bacteroidetes* (~19.9%), *Actinobacteria* (~4.1%) and *Chloroflexi* (~1.0%) (Figure 3A). At the genus level, the results showed that 20 dominant genera (*Moraxella, Pseudomonas, Lactobacillus, Prevotella, Bacteroides, Megasphaera, Streptococcus, Rothia, Allobaculum, Blautia, Oscillospira, Kingella, Halomonas, Sutterella, Faecalibacterium, Prevotella, Ochrobactrum, Ruminococcus, Akkermansia*, and *Propionibacterium*), which constituted over 1% of the total sequences on average, were present in the microbial communities (Figure 3B). The results indicated that the microbial relative abundance in samples exposed to ammonia at 25 ppm was significantly different than those in the other groups at both the phylum and genus levels.

The article "The Variation of Nasal Microbiota Caused by Low Levels of Gaseous Ammonia Exposure in Growing Pigs" was retracted in 2025. Reasons: unreliable results or conclusions; concerns about the article.

**Figure 3:** Alterations in nasal microbial taxonomic compositions with the low levels of gaseous ammonia exposure. **(A)** Graph represents the OTUs at different taxonomical levels: phylum (*n* = 12). **(B)** Graph represents the OTUs at different taxonomical levels: genus (*n* = 12). **(C)** The change in the relative abundance of genus Moraxella, Pseudomonas, Lactobacillus, Prevotella, Bacteroides, Streptococcus with the low levels of gaseous ammonia exposure. Metastats analysis was applied to identify the significantly differentially abundant genera among groups. Different letters above the bars denotes significantly differentially abundant genera among groups. (Data are mean ± SD; and *P < 0.05; **P < 0.01).

To evaluate how the nasal microbial taxonomic compositions at the phylum and genus level altered as levels of gaseous ammonia changed, a Metastat analysis was performed to identify the differentially abundant phyla and genera among groups. We chose to show the abundance distribution of the first 20 classification units with the most significant differences between groups (*n* = 12) (Figure S3). All 20 abundant genera accounted for over 98.3% of the total sequences in the samples. Among the 20 genus units, there was a significant change in 6 genera (*Moraxella, Pseudomonas, Lactobacillus, Prevotella, Bacteroides*, and *Streptococcus*) under different low levels of gaseous ammonia exposure. The relative abundances of 4 genera (*Pseudomonas, Lactobacillus, Prevotella, Bacteroides*) significantly decreased at 25 ppm compared with those in the other groups, while the microbial community showed significant increases in the relative abundance of only two genera (*Moraxella* and *Streptococcus*) at 25 ppm (Figure 3C).

The article "The Variation of Nasal Microbiota Caused by Low Levels of Gaseous Ammonia Exposure in Growing Pigs" was retracted in 2025. Reasons: unreliable results or conclusions; concerns about the article.

### Identification of Nasal Microbiota Associated With Metabolic Function With Low Levels of Gaseous Ammonia Exposure

To further investigate the nasal microbiota associated with metabolic function development with low levels of gaseous ammonia exposure in pigs, the PICRUSt approach was used to analyze the KEGG pathway compositions in nasal microbiota populations. The KEGG pathway analyses resulted in annotations related to cellular processes, environmental information processing, genetic_information_processing diseases, metabolism, and organismal systems. According to the results of cellular processes (Figure 4A), the relative abundances of the genes involved in cell motility at 20 and 25 ppm were significantly decreased compared with those in the other groups. The results of environmental information processing showed a significant decrease in the relative abundances of the genes involved in signal transduction and membrane transport when pigs were exposed to gaseous ammonia at 25 ppm and showed a decreasing trend with increasing ammonia concentrations (Figure 4B). According to the results of genetic_information_processing, the relative abundances of the genes involved in translation, replication and repair and folding, sorting and degradation at 0 and 25 ppm significantly increased compared with those in the other groups (Figure 4C).

**Figure 4:** Identification of Nasal Microbiota Associated with Metabolic function with the low levels of gaseous ammonia exposure. **(A)** KEGG pathways compositions in nasal microbiota populations: cellular processes. **(B)** KEGG pathways compositions in nasal microbiota populations: environmental information processing. **(C)** KEGG pathways compositions in nasal microbiota populations: genetic_information_processing. **(D)** KEGG pathways compositions in nasal microbiota populations: diseases. **(E)** KEGG pathways compositions in nasal microbiota populations: metabolism. **(F)** KEGG pathways compositions in nasal microbiota populations: organismal systems. The ordinate is the relative abundance of each functional group in each group. This is shown in the form of a violin diagram combined with a box chart. The violin diagram can visually display the distribution of the data, the “violin” (The width of the sample, indicating that the corresponding amount of the corresponding sample); box chart border represents the upper and lower quartile spacing (Interquartile range, IQR), horizontal line Represents the median, the upper and lower tentacles represent the upper and lower quartile 1.5 times IQR range, the symbol “•” that over the range of extreme values. The graph can be used to compute the results of the Metastats difference significance analysis.

The article "The Variation of Nasal Microbiota Caused by Low Levels of Gaseous Ammonia Exposure in Growing Pigs" was retracted in 2025. Reasons: unreliable results or conclusions; concerns about the article.

As for organismal systems, the relative abundances of the genes involved in the immune system, endocrine system, and circulatory system at the 25 ppm ammonia level significantly increased compared with those in the other groups and showed an increasing trend in the digestive system and excretory system with increasing gaseous ammonia levels. In contrast, the microbial community showed a significant decrease in environmental adaptation at 25 ppm and a decreasing trend in the nervous system with increasing ammonia concentrations (Figure 4F).

For the relative abundances of the genes involved in diseases and metabolism (Figures 4D,E), the results showed an increasing trend in immune system diseases and cancer with the increase of ammonia concentration and a significant increase in neurodegenerative diseases at the 25 ppm level compared with the other groups. Genes involved in metabolic diseases decreased with increasing ammonia levels. In addition, the microbial community also showed a shift in metabolism with the levels of gaseous ammonia exposure. The results showed an increasing trend in the relative abundances of genes related to the metabolism of nucleotide terpenoids and polyketides, cofactors and vitamins, lipid, and amino acids, while energy and carbohydrate metabolism genes decreased with the increase of gaseous ammonia levels.

### Effect of Gaseous Ammonia Exposure on the Respiratory Mucosal Barrier, Growth Performance, and the Quantity of *Moraxella* and *Streptococcus* in Growing Pigs

It was demonstrated that the nasal microbiota in growing pigs shifts with the increase in low-level gaseous ammonia exposure according to the above results. However, how do low levels of gaseous ammonia exposure affect the health of pigs? We evaluated the effect of gaseous ammonia exposure on the respiratory mucosa, growth performance and the quantity of *Moraxella* and *Streptococcus* in growing pigs.

We first tested the effect of ammonia on growth performance and immunological measures of growing pigs. The results of growth performance analyses are shown in Figure 5A. No significant differences were observed with regard to ADF and FCR at all ammonia exposure levels from 0 to 25 ppm. However, increasing the concentration of ammonia contributed to a decrease in the ADG of growing pigs (linear, P < 0.05), reached its lowest value at 25 ppm. Additionally, regarding clinical findings, the increasing concentration of ammonia contributed to more severe clinical signs, such as coughing, sneezing difficult breathing and conjunctivitis (Table 1). The effect of ammonia concentration on the blood biochemical indices of growing pigs is shown in Table 2. Blood ammonia, BUN, SOD, T-AOC, LDH, and AST had extremely significant linear correlations with ammonia concentration (linear effect P < 0.01). Blood ammonia and ammonia concentrations were significantly positively correlated (linear effect P < 0.01). There was a significant positive correlation between BUN and ammonia concentration (linear effect P < 0.01). The levels of BUN in the 15–25 ppm groups were significantly higher than those in the 0 and 5 ppm group (*P* < 0.05). SOD and T-AOC were significantly negatively correlated with the increase in ammonia concentration (linear effect *P* < 0.01). The SOD contents in the 10–25 ppm groups were significantly lower than that in the 0 and 5 ppm group (*P* < 0.05). The T-AOC values were significantly lower in the 15–25 ppm groups than those in the 0 and 5 ppm group (*P* < 0.05). LDH and AST showed a highly significant positive correlation with increasing concentrations of ammonia (linear effect *P* < 0.01). LDH levels in the 20–25 ppm groups were significantly higher than those in the 0 and 5 ppm group (*P* < 0.05), and AST levels in the 10–25 ppm groups were significantly higher than those in the 0 ppm group (*P* < 0.05).

The article "The Variation of Nasal Microbiota Caused by Low Levels of Gaseous Ammonia Exposure in Growing Pigs" was retracted in 2025. Reasons: unreliable results or conclusions; concerns about the article.

**Figure 5:** Effect of gaseous ammonia exposure on respiratory mucosal barrier and growth performance of growing pigs **(A)** Effect of ammonia on growth performance of growing pigs. **(B)** Effects of different concentrations of ammonia on levels of immune globulin in growing pigs. **(C)** Effects of different concentrations of ammonia on the morphology of tracheal mucosa in growing pigs. **(D)** Effects of different concentrations of ammonia on the lung tissue morphology of growing pigs. Values with no common superscripts means significant difference (*P* < 0.05).

**Table 1:** Effect of gaseous ammonia exposure on clinical findings and macroscopic lesions of pigs^a^.

**Item**	**Ammonia concentration, ppm**					
	**0**	**5**	**10**	**15**	**20**	**25**
Coughing pigs per treatment	0	1	3	4	6	15
Sneezing pigs per treatment	0	0	2	4	6	9
Difficult breathing pigs per treatment	0	0	1	2	7	14
Pinkeye pigs per treatment	0	0	0	0	2	7

a *A total of 120 growing pigs (6 treatment, 20 pigs per treatment) with an average initial BW of 30.2 ± 1 kg. Nasal swab samples were randomly collected from 72 pigs (n = 12)*.

**Table 2:** Effects of different concentration ammonia on blood biochemical index of growing pigs.

**Biochemical index**	**Ammonia concentration, ppm**						**SEM**	**Contrast^1^**	
	**0 ppm**	**5 ppm**	**10 ppm**	**15 ppm**	**20 ppm**	**25 ppm**		**L**	**Q**
Blood ammoni(μmol/L)	144.38^b^	146.51^b^	155.36^b^	159.07^b^	173.63^ab^	195.19^a^	5.54	<0.01	0.272
BUN(mmol/L)	2.69^d^	2.89^d^	3.34^cd^	3.62^bc^	4.09^ab^	4.18^a^	0.14	<0.01	0.374
SOD(U/L)	171.35^a^	162.32^a^	142.21^b^	139.20^b^	125.74^c^	119.72^c^	4.12	<0.01	0.153
T-AOC(μmol/L)	1.58^a^	1.56^a^	1.44^ab^	1.25^bc^	1.07^c^	1.00^c^	0.07	<0.01	0.750
LDH(U/L)	499.61^c^	483.14^c^	471.11^c^	531.83^bc^	560.12^b^	664.99^a^	19.87	<0.01	0.017
AST(U/L)	4.01^d^	4.56^d^	6.52^c^	10.55^b^	9.89^b^	12.77^a^	0.79	<0.01	0.019

1 *Contrast: L means linear effect, Q means quadratic effect. Values with no common superscripts means significant difference (P < 0.05)*.

The article "The Variation of Nasal Microbiota Caused by Low Levels of Gaseous Ammonia Exposure in Growing Pigs" was retracted in 2025. Reasons: unreliable results or conclusions; concerns about the article.

The effects of different concentrations of ammonia on the levels of immunoglobulin in growing pigs are shown in Figure 5B. IgG levels were significantly linearly related to the increase in ammonia concentrations (linear, *P* < 0.01). The IgG levels of the 20–25 ppm groups were significantly lower than the other groups (*P* < 0.05). IgA and IgM levels showed a highly significant linear correlation with the change in ammonia concentration (linear, *P* < 0.01). The IgA and IgM levels in the 20–25 ppm groups were significantly lower than the other groups (*P* < 0.05).

We next tested the effect of ammonia on the respiratory mucosal barrier of growing pigs. The effects of different ammonia concentrations on the expression of trachea-related genes in growing pigs are shown in Table 3. Muc5b gene expression was linearly correlated with ammonia concentration (linear effect *P* < 0.05). The expression of mucin in the 20 ppm group was the highest and was significantly higher than that in the 0 and 5ppm group (*P* < 0.05). There was a significant negative correlation between the expression of the Claudin-1 gene and ammonia concentration (linear, *P* < 0.05). The expression of Claudin-1 reached its maximum in the 0 ppm group and was significantly lower in the 25 ppm group than in the 0 and 5 ppm group (*P* < 0.05). The expression of the caspase-3 gene was significantly and linearly correlated with ammonia concentration (linear, *P* < 0.01). The expression level was highest in the 25 ppm and was significantly increased in the 20–25 ppm groups (*P* < 0.05).

**Table 3:** Effects of different concentration ammonia on trachea-related gene expression of growing pigs.

**Measured gene**	**Ammonia concentration, ppm**						**SEM**	**Contrast^1^**	
	**0 ppm**	**5 ppm**	**10 ppm**	**15 ppm**	**20 ppm**	**25 ppm**		**L**	**Q**
muc5b	0.64^c^	0.77^c^	1.25^bc^	1.40^b^	2.42^a^	2.37^a^	0.25	0.016	0.926
Claudin-1	1.62^a^	1.57^a^	1.52^ab^	1.33^b^	1.11^c^	0.85^d^	0.10	0.014	0.568
caspase-3	0.48^c^	0.52^c^	0.68^c^	1.04^b^	1.19^ab^	1.38^a^	0.11	<0.01	0.817

1 *Contrast:L means linear effect,Q means quadratic effect. Values with no common superscripts means significant difference (P < 0.05)*.

The article "The Variation of Nasal Microbiota Caused by Low Levels of Gaseous Ammonia Exposure in Growing Pigs" was retracted in 2025. Reasons: unreliable results or conclusions; concerns about the article.

The effects of different concentrations of ammonia on the morphology of the tracheal mucosa of growing pigs are shown in Figure 5C. Ammonia treatments at 0–10 ppm resulted in a relatively intact tracheal mucous membrane structure. In the 15–20 ppm ammonia environment, the cilia of the tracheal mucosa were moderately deteriorated. In the presence of 25 ppm ammonia, the structure of the tracheal mucosal layer was severely deformed, and the columnar cilia of the pseudostratified layer were also largely absent. The influence of different concentrations of ammonia on the lung tissue morphology of growing pigs is shown in Figure 5D. Negative effects of 0 ppm~25 ppm ammonia gas concentrations on the tracheal mucosa of pigs continued to increase. The alveolar cavity was visible after 0–10 ppm ammonia stimulation; however, there was a large infiltration of inflammatory cells in the alveoli under 25 ppm exposure, and the alveolar spaces were reduced.

As the genera *Moraxella* and *Streptococcus* were increased in the of 25 ppm group, we quantified these two bacterial species in the nasal swabs by using quantitative real-time PCR analysis. Species-specific PCR primers are listed in Table 4. The results are shown in Table 5. Increasing concentrations of ammonia increased both the number of *Moraxella catarrhalis* and *Streptococcus pneumoniae*, and the number of both bacteria in pigs from the 20 and 25 ppm groups was significantly higher than those from the other groups (linear, *P* < 0.05), which was consistent with previous results for this genus.

**Table 4:** Primers used for several microflora.

**Bacteria**	**Primer**	**Sequence (5^**′**^-3^**′**^)**	**References**
*Moraxella catarrhalis*	Forward: UspA1-F	GCGTCTGC ACAACAACCAAA	(Tao et al., 2017)
	Reverse: UspA1-R	TGTCGCCTAT GGCTTCGTTT	
*Streptococcus pneumoniae*	Forward: Dp1	CTGTGGCTT AACCATAGTAG	(El Aila et al., 2010)
	Reverse: Dp2	CTAGCACTCAT CGTTYACA	

**Table 5:** Quantitative real-time PCR analysis of total *Moraxella catarrhalis, Streptococcus pneumoniae* in nasal swab samples [Log 10 (copies/g wet weight)]^a^.

**Item**	**Ammonia concentration, ppm**						**SEM**	***P*****-value**	
	**0**	**5**	**10**	**15**	**20**	**25**		**Linear**	**Quadratic**
*Moraxella- catarrhalis*	7.49^a^	7.75^a^	7.84^a^	8.75^ab^	10.51^b^	13.92^c^	0.32	<0.01	0.147
*Streptococcus pneumoniae*	5.08^a^	5.25^a^	6.48^a^	7.56^ab^	8.49^b^	10.37^c^	0.42	<0.01	0.097

a *A total of 120 growing pigs (6 treatment and 20 pigs per treatment) with an average initial BW of 30.2 ± 1kg. Nasal swab samples were randomly collected from 72 pigs (n = 12)*.

*Contrast:L means linear effect,Q means quadratic effect. Values with no common superscripts means significant difference (P < 0.05)*.

The article "The Variation of Nasal Microbiota Caused by Low Levels of Gaseous Ammonia Exposure in Growing Pigs" was retracted in 2025. Reasons: unreliable results or conclusions; concerns about the article.

## Discussion

Pigs reared in intensive production systems are continuously exposed to gaseous ammonia released during the microbial degradation of their excrement (Hamilton et al., 1998). Recently, pig farming was found to have an extensive effect on the nasal microbiota of humans and pigs, and studies have suggested that the nasal microbiota of humans and pigs are intimately connected with respiratory diseases (Kraemer et al., 2018). Current ammonia levels within commercial pig buildings are not extremely high and typically in the region of 10 to 25 ppm (Costa et al., 2003). However, it was reported that even low levels of gaseous ammonia have toxic effects on the respiratory tract of pigs. A previous study found that *Bacillus pasteurii* was significantly increased in piglets exposed to 20 ppm gaseous ammonia and caused atrophic rhinitis (Hamilton et al., 1998). This indicates that ammonia can affect respiratory mucosal microbiota, and the harmful bacteria in the microbiota may damage animal health after becoming the dominant population. The nasal cavity is part of the mucosal system of the upper respiratory tract, and its microbial composition shifts with changes in the environment. Therefore, the nasal microbial composition can reflect the entire respiratory tract composition of microorganisms (Yan et al., 2013; Zeineldin et al., 2017). Thus, the aims of this article were to describe the effect of low concentrations of ammonia on the respiratory tract and nasal microbiota in growing pigs.

In this study, by using controlled environmental chambers, we were able to control gaseous ammonia concentrations from 0–25 ppm accurately in the chambers. The environmental control box in this experiment was used for the automatic and accurate control of various gases. It has been compared with the traditional corral, and it is able control single environment variables and various environmental factors (Murphy et al., 2012). The present study showed that the number of OTUs in the 20 and 25 ppm groups were significantly lower than those in the other groups. Similarly, the alpha diversity of the nasal microbial community was also significantly decreased at concentrations of 20–25 ppm ammonia. Furthermore, beta diversity analysis showed significant differences in pigs exposed to different levels of ammonia, especially those exposed to 20–25 ppm. The reason may be an alkaline environment in the nasal cavity caused by the higher ammonia concentration damage, which affects the colonization of acidophilic bacteria (Valdes et al., 2009).

Consistent with previous studies on pigs (Slifierz et al., 2015; Correa-Fiz et al., 2016), this study demonstrated that *Proteobacteria, Firmicutes*, and *Bacteroidetes* were the three most dominant phyla in the nasal bacterial communities of piglets. The results obtained in the study based on the nasal microbiota in pigs with Glässer's disease indicated that the *Proteobacteria, Firmicutes*, and *Bacteroidetes* were the most prevalent phyla, suggesting similarities between the pigs exposed to ammonia and Glässer's disease (Correa-Fiz et al., 2016). Glässer's disease is often accompanied by pneumonia and respiratory disease, which may be caused by high levels of ammonia exposure in pig farming (Beskow et al., 2010). This study also showed that 20 abundant genera accounted for over 98.3% of the total sequences in the samples. Among them, the dominant bacterial communities were *Moraxella, Pseudomonas, Lactobacillus, Prevotella, Bacteroides*, and *Streptococcus*. Of note, the relative abundances of *Moraxella* and *Streptococcus* were significantly higher than those in the other groups, while the relative abundances of 4 phyla (*Pseudomonas, Lactobacillus, Prevotella*, and *Bacteroides*) were significantly decreased in the 25 ppm group compared with the other groups. Previous studies have shown that *Moraxella* and *Streptococcus* are common pathogenic bacteria in lung tissues of patients with pneumonia (Riise et al., 2000). This suggests that a large number of *Moraxella* present in the nasal cavity may enter the alveoli during respiration, causing inflammation in the lungs and leading to obstructive pneumonia. In addition, *Streptococcus* includes suppurative *Streptococcus, Streptococcus pneumonia*, and other harmful bacteria (Riise et al., 2000). These two pathogenic bacteria showed a significant increase in the nasal cavity of pigs exposed to 25 ppm ammonia, and these alterations in nasal microbiota may cause lung pathology in pigs (Gutbier et al., 2015), which was consistent with the results of lung tissue morphology in this research. *Lactobacillus* is a beneficial bacteria to the intestines of pigs and produces organic acids that help the large intestine use fiber (Smith, 2006). However, the effect of *Lactobacillus* on the respiratory tract of pigs is unclear, but reports have indicated that *Lactobacillus* in the respiratory tract can inhibit the growth and reproduction of *E. coli* and other harmful bacteria (Hang et al., 2009). In this experiment, *Lactobacillus* was the second most dominant genera in the 0–15 ppm groups and was significantly higher than the *Lactobacillus* in the 20–25 ppm treatment groups. This may be due to the high ammonia concentration causing a high pH value, inhibiting the growth and colonization of *Lactobacillus*; moreover, populations of harmful bacteria inhibit the growth of the *Lactobacillus* genera (Gandhi and Shah, 2014).

The article "The Variation of Nasal Microbiota Caused by Low Levels of Gaseous Ammonia Exposure in Growing Pigs" was retracted in 2025. Reasons: unreliable results or conclusions; concerns about the article.

In addition to the development of the nasal microbiota, the functional maturation of the microbiome was also assessed using PICRUSt (Langille et al., 2013; Buffie et al., 2015). The present study analyzed the KEGG pathway compositions in nasal microbiota populations, resulting in the identification of genes related to cellular processes, environmental information processing, diseases, metabolism, and organismal systems. The results of cellular processes showed that the relative abundances of the genes involved in cell motility were significantly decreased in the 20 and 25 ppm groups compared with the other groups, suggesting that even at low levels of gaseous ammonia exposure, cell motility may be inhibited. Furthermore, in organismal systems, nasal microbiome gene related to the immune system, endocrine system, and circulatory system were significantly increased in the 25 ppm group compared with the other groups. In contrast, the microbial community of the 25 ppm group showed a significant decrease in environmental adaptation genes and a decreasing trend in nervous system genes with increasing ammonia concentration. This may be due to the stress response caused by the ammonia stimulation (Xu and Zheng, 2018), consistent with our results regarding immunological measures. Moreover, for the relative abundances of the genes involved in diseases and metabolism, nasal microbiome genes involved in immune system diseases and cancer increased with the increase in ammonia levels, and genes of neurodegenerative diseases significantly increased in the 25 ppm group. These results are consistent with previous studies that indicated that high levels of ammonia can change the pH of blood, which stimulates the brain nerve center and causes neurodegenerative diseases (Rama Rao et al., 2003). In addition, the microbial community also showed a shift in metabolism with the levels of gaseous ammonia exposure. The increase of ammonia concentration increased the lipid and amino acid metabolism but decreased the energy and carbohydrate metabolism of pigs, which may indicate that lipid and amino acids were preferentially utilized over carbohydrates in pigs exposed to low levels of gaseous ammonia.

Previous studies have examined the impact of the exposure to ammonia gas on the upper respiratory system and growth rates of pigs. It was found that aerial ammonia decreased the growth of young (8-wk-old) pigs, and the reduction in average daily gain compared with controls was 12, 30, and 29% for groups exposed to 50, 100, and 150 ppm ammonia, respectively (Drummond et al., 1980). Acute inflammatory responses were also observed in the tracheal epithelium of pigs exposed to 100 and 150 ppm atmospheric ammonia but not in controls or pigs subjected to 50 ppm atmospheric ammonia (Costa et al., 2003). Nevertheless, atmospheric ammonia concentrations of 50, 100 and 150 ppm are inappropriate to study since the range is too high for the useful comparison to production conditions. Our results showed that increasing ammonia concentrations higher than 10 ppm increased blood ammonia and urea nitrogen concentrations and decreased the antioxidant ability of pigs, concentrations higher than 15 ppm affected the expression of genes related to the integrity of the trachea structure, concentrations higher than 20 ppm reduced the levels of immunoglobulins in the mucosa of pig trachea, and concentrations higher than 25 ppm significantly damaged tracheal mucosa cilium and alveoli and decreased growth performance. These results indicated different sensitivities of genes, tissues and bodies to ammonia. At ammonia concentrations <25 ppm, a large number of inflammatory cells were found in the alveolar cavity, and severe hyperemia of the lung tissue may have been associated with the nasal microbiota analysis results. A large amount of *Moraxella* and *Streptococcus* in the nasal cavity may have caused an inflammatory response in the lungs of the 25 ppm group, while the decrease in pig performance may be due to inflammation and injury of the lung tissue. In addition, as a result of the increase in ammonia to 25 ppm, harmful bacteria become dominant, and the colonization of beneficial bacteria may be affected. The imbalance of nasal microbiota will lead to respiratory mucosal immune function disorders in the respiratory tract (Korten et al., 2018). Here, it was demonstrated that ammonia concentrations higher than 20 ppm decreased the abundance of microbiota in the nasal cavity of growing pigs and increased the colonization of harmful bacteria, which may lead to respiratory diseases in pigs.

The article "The Variation of Nasal Microbiota Caused by Low Levels of Gaseous Ammonia Exposure in Growing Pigs" was retracted in 2025. Reasons: unreliable results or conclusions; concerns about the article.

In summary, the present study revealed the composition of the nasal microbiota communities associated with low levels of gaseous ammonia exposure. This study also indicted that the threshold concentration of ammonia in pig farming is 20 ppm. The results of this study indicated that gaseous ammonia in the pig farming environment significantly changed the nasal microbiota communities, and high concentrations of ammonia may cause respiratory damage and even pneumonia by affecting the colonization rates of harmful bacteria and beneficial bacteria. Thus, our study may facilitate the development of animal models for research on the nasal microbiota, as well as for the health of human beings and pigs.

Nevertheless, there were some limitations in this study. The removal of feces hourly reduced the exposure to gastrointestinal flora, which may affect the composition of the nasal microbiota. In addition, due to the artificial environment, it was difficult to determine if similar results would be found in pigs living on farms. Ideally, performing OTU analyses for farmed pigs exposed to high and low levels of ammonia would result in a better correlation between the analysis and real-world applications.

## Author Contributions

TW and FH designed the research. TW, QH, WY, YS, and JL conducted the research. TW and QH analyzed the data. TW wrote the manuscript. All authors read and approved the final version of the manuscript.

### Conflict of Interest Statement

The authors declare that the research was conducted in the absence of any commercial or financial relationships that could be construed as a potential conflict of interest.
